# Photoactivatable Hsp47: A Tool to Regulate Collagen Secretion and Assembly

**DOI:** 10.1002/advs.201801982

**Published:** 2019-02-28

**Authors:** Essak S. Khan, Shrikrishnan Sankaran, Julieta I. Paez, Christina Muth, Mitchell K. L. Han, Aránzazu del Campo

**Affiliations:** ^1^ INM‐Leibniz Institute for New Materials Campus D2 2 ,66123 Saarbrücken Germany; ^2^ Chemistry Department Saarland University 66123 Saarbrücken Germany

**Keywords:** collagen deposition, KDEL receptor‐mediated endocytosis, noncanonical amino acid incorporation, photoactivation, Hsp47

## Abstract

Collagen is the most abundant structural protein in mammals and is crucial for the mechanical integrity of tissues. Hsp47, an endoplasmic reticulum resident collagen‐specific chaperone, is involved in collagen biosynthesis and plays a fundamental role in the folding, stability, and intracellular transport of procollagen triple helices. This work reports on a photoactivatable derivative of Hsp47 that allows regulation of collagen biosynthesis within mammalian cells using light. Photoactivatable Hsp47 contains a non‐natural light‐responsive tyrosine (o‐nitro benzyl tyrosine (ONBY)) at Tyr383 position of the protein sequence. This mutation renders Hsp47 inactive toward collagen binding. The inactive, photoactivatable protein is easily uptaken by cells within a few minutes of incubation, and accumulated at the endoplasmic reticulum via retrograde KDEL receptor‐mediated uptake. Upon light exposure, the photoactivatable Hsp47 turns into functional Hsp47 in situ. The increased intracellular concentration of Hsp47 results in stimulated secretion of collagen. The ability to promote collagen synthesis on demand, with spatiotemporal resolution, and in diseased state cells is demonstrated in vitro. It is envisioned that photoactivatable Hsp47 allows unprecedented fundamental studies of collagen biosynthesis, matrix biology, and inspires new therapeutic concepts in biomedicine and tissue regeneration.

## 1 Introduction

Collagen is a major component of the extracellular matrix, and the most abundant structural protein for the mechanical integrity of tissues.^1^ A collagen molecule consists of a characteristic triple helix formed by three α‐chains. In vivo, collagen molecules self‐assemble to form collagen fibrils, beaded filaments, or network structures depending on the collagen type. This assembly is the basis for achieving tissue‐specific mechanical properties: rigid bone, compliant skin, or gradient mechanics in cartilage tissue.^2^ The dynamics of collagen synthesis and deposition plays a crucial role in biological processes such as embryogenesis^3^ and tissue regeneration,^4^ while it gets dysregulated in pathologies like brittle‐bone disease,^5^ fibrosis or tumor formation.^6^ As the main underlying supportive structure for cells, the deposition of collagen typically precedes and guides the development of tissue architectures. For instance, in lungs, salivary and mammary glands, the spatial distribution and density of predeposited collagen directs the formation of branched tissue configurations.^7^ In spinal cord^8^ and arterial injuries,^9^ it has been shown that initial collagen deposition by the underlying fibroblasts is vital for the remodeling of these tissues, resulting in their healing. While extensive efforts have been made to understand and replicate these phenomena, the existing molecular strategies to probe collagen deposition require the use of chemicals such as ascorbate,^10^ growth factors like TGF‐β and FGF, and genetic modifications.^11^ However, these molecules interfere with many cellular processes and do not allow localized manipulation at single cell level.^12^ The possibility to regulate collagen deposition specifically, on demand and eventually in a spatially confined manner would allow precise studies in collagen‐related cellular processes for fundamental and therapeutic purposes.

In this study, we have taken the first steps in this direction by developing and testing a molecular tool that enables spatiotemporal manipulation of collagen synthesis and deposition using light irradiation as remote trigger. We targeted a molecular chaperone, Hsp47 (Heat shock protein 47) that is known to be vital for collagen biosynthesis within cells.^12^, ^13^ It is a highly conserved, 47‐kDa endoplasmic reticulum (ER)‐resident protein known to bind collagen types I to V (and possibly others),^14^ and plays a fundamental role in the folding, stability and intracellular transport of procollagen triple helices.[[qv: 13c]] Procollagen is inherently unstable at physiological temperature and prone to intracellular degradation. Hsp47 protects it by stabilizing the triple helix, thereby providing a quality control mechanism for correct helical folding and assembly while simultaneously preventing premature aggregation of the helices.^15^ Constitutive expression levels of Hsp47 strongly correlate with the amounts of collagen being synthesized in the corresponding cells.[[qv: 13d,16]] For example, expression of Hsp47 is upregulated during the progression of various fibrotic lesions.^17^ Studies have shown that suppression of Hsp47 expression can reduce accumulation of collagen and can delay the progression of fibrotic diseases in experimental animal models.^18^ Alternatively, knocking out its expression in mouse embryos has been found to result in a lethal phenotype.^19^ Collagen biosynthesis therefore strongly depends on the correct expression and function of Hsp47, and hence can be altered by interfering with Hsp47 activity. We hypothesized that a light‐activatable version of Hsp47 would allow us to remotely control the biosynthesis and, subsequently, the deposition of collagen.

Controlling intracellular protein function by light is possible by introducing photoresponsive non‐natural amino acids at the active site in the protein structure.^20^ Hsp47 binds collagen at its typical Gly‐Xaa‐Yaa amino acid repeats. Reported literature[[qv: 13a]] has shown that when Arg occupies the Yaa position, the Asp385 rest in Hsp47 binds to the collagen triple helix strand by forming a salt bridge. Further stabilization of this complex is provided through Tyr383 and Leu381 through hydrophobic interactions. In its triple helical form, collagen forms a complex with Hsp47 with a total solvent‐accessible surface area of 1000 ± 150 Å^2^ buried between them, indicating tight interactions within the binding site.[[qv: 13a]] Interestingly, while mutations in Hsp47's Asp385 and Leu381 seem to reduce its affinity with collagen, mutations in Tyr383 were shown to completely inhibit the interaction, indicating that this residue plays a major role in the binding.[[qv: 13a,17a]] Therefore, this position was identified as suitable site for the introduction of a photoactivatable rest to control Hsp47 binding to collagen with light. Luckily, synthetic tools to incorporate the non‐natural light‐responsive tyrosine (o‐nitro benzyl tyrosine (ONBY)) amino acid on recombinant proteins have been previously developed.^21^ It has been shown that replacement of Tyr by ONBY in Tyr‐stabilized protein‐protein or protein‐DNA complexes lead to destabilization of the complex via steric hindrance and disruption of hydrophobic interactions due to the polar nitro group.^21^ We hypothesized that a similar effect would occur when replacing Tyr383 by ONBY in Hsp47 structure to obtain the photoactivatable variant H_47Y<ONBY_.

The delivery of recombinant proteins from the medium into the ER of cells was considered a challenge for our objective. Initially, microinjection of the protein into the ER was planned.^22^ However, during the course of this study a KDEL receptor‐mediated endocytosis mechanism capable of transporting proteins containing an ER retention motif (KDEL) to the ER was observed. By including KDEL motif in the recombinantly synthesized H_47<ONBY_, the possibility to deliver it to the ER by simple incubation was attempted and successfully achieved. Using this strategy, collagen production and deposition in disease‐state Hsp47‐knocked out fibroblast cells was realized. This article demonstrates on demand deposition of collagen by activation of a new molecular tool with spatiotemporal control.

## 2 Results and discussion

### 2.1 Synthesis and Purification

A previously developed Hsp47 gene coding for residues 36–418 was used.[[qv: 13a]] In order to improve Hsp47's solubility for heterologous expression in *E. coli*, an enhanced green fluorescent protein (EGFP) was genetically fused to its N‐terminal.^23^ This approach led to a significant increase in the synthesis yield (Table S1, Supporting Information). A StrepII‐tag was introduced at the C‐terminal for affinity purification. This derivative of Hsp47 was successfully obtained in 207.8 µg yield from 200 mL culture, as confirmed by absorbance with UV–vis spectrophotometer, and was named H_47N_ (N refers to native). The o‐nitrobenzyl tyrosine (ONBY) rest was incorporated at 383rd position via a previously established bacterial‐engineering strategy^24^ (see details in Figure S1 in the Supporting Information). An amber codon mutation TAG incorporated ONBY specifically at the 383rd position. This Hsp47 derivative was named H_47Y<ONBY_.

In order to confirm the incorporation of ONBY, synthesis in the presence or absence of ONBY in the medium before induction was performed. In the presence of ONBY, the full protein would be expressed, whereas in the absence of ONBY, translation should terminate at the 383rd position and the StrepII‐tag would not be included. Agarose beads with affinity toward the StrepII‐tag were incubated with small amount of cleared lysates and purified Hsp47 control variants. The agarose beads became fluorescent within 5 mins when incubated with H_47Y<ONBY_, indicating that the StrepII‐tag had been incorporated at the C‐terminus (ONBY present) whereas no fluorescence was observed in truncated version having no StrepII‐tag (**Figure** **1**b). The clear lysates were purified using StrepII‐tag affinity purification and screened to affirm the presence of StrepII‐tag. Western Blot was performed labeling StrepII‐tag using Alexa488‐Streptavidin after affinity purification which showed a clear fluorescent band when ONBY was present during synthesis, and no fluorescence was observed in the truncated version (Figure 1c). This result confirmed the incorporation of ONBY to H_47Y<ONBY_. The yield of the synthesis was 43.56 ng from 200 mL culture. Two additional mutants of H_47N_ were developed as control proteins for further experiments: i) H_47Y<R,_ with Tyrosine mutated to Arginine at 383rd position as an inactive version of H_47N_.[[qv: 13a]] ii) H_47KDEL_ where the KDEL sequence at C terminus of H_47N_ was deleted, thereby preventing retrograde delivery of the protein into the ER. The yields of all the variants are included in Table S1 in the Supporting Information.

**Figure 1:** Structure and characterization of photoactivatable Hsp47 (H_47Y<ONBY_). a) Scheme showing the structure of Hsp47: collagen peptide interaction^19^ and the photocleavage reaction of ONBY. b) Microscopy images (merged phase contrast and epifluorescence green channels) of StrepII‐tagged agarose beads incubated with supernatant of different Hsp47 variants showing the presence or absence of StrepII‐tag in the protein structure (scale bar 100 µm). c) 12% sodium dodecyl sulfate (SDS) PAGE gel and Western Blot of purified H_47Y<ONBY_ (truncated and full) stained with Alexa 488 conjugated Streptavidin (blue).

### 2.2 Photoactivatable Hsp47 Specifically Binds to Collagen Upon Activation

In order to verify the affinity of the different Hsp47 variants (H_47N_, H_47Y<ONBY_, H_47Y<R_, H_47KDEL_) for collagen, the obtained proteins were incubated with micropatterns of collagen I on a substrate (see Experimental Section for details)^25^ and imaged by fluorescence microscopy. H_47N_ and H_47KDEL_ showed fluorescence bands (green fluorescence due to EGFP tagged constructs) indicating interaction to collagen, whereas H_47Y<ONBY_, the negative control H_47Y<R_, and the EGFP did not bind to collagen (**Figure** **2**a).Light irradiation of the H_47Y<ONBY_ solution during incubation (in situ activation upon 10 sec exposure at 365 nm) lead to appearance of fluorescence bands. This result demonstrates that photochemical activation of H_47Y<ONBY_ renders functional Hsp47 (H_47Y<ONBY_ *_hv_*), able to bind to collagen. Native PAGE‐western blot analysis confirmed these results (Figure 2b). Colocalization of fluorescent antibody labeled bands of collagen and H_47N_ or light‐activated H_47Y<ONBYhv_ was observed. Conversely, H_47Y<ONBY_, H_47Y<R_ and EGFP did not colocalize with the collagen band, demonstrating no collagen binding.

**Figure 2:** Photoactivatable Hsp47 affinity and function assay. a) Schematic of affinity test using a protein micropattern designed to detect affinity of Hsp47 and its different variants to collagen. The corresponding fluorescence image of the binding assay shows the obtained results. b) Native PAGE Western Blot of rat‐tail collagen Type 1 (200 µg mL^−1^, 0.6 × 10^−6^ m) mixed with H_47N_, H_47Y<R_, H_47Y<ONBYhv_, or H_47KDEL_ (1.2 × 10^−6^ m), demonstrating colocalization of Hsp47 variants with collagen in binding assays. c) Fibrillogenesis assay by turbidimetry measurements of collagen (200 µg mL^−1^, 0.6 × 10^−6^ m) mixed with H_47N_, H_47Y<R_, H_47Y<ONBYhv_, or H_47KDEL_ (1.2 × 10^−6^ m) at molar ratio 2:1(Hsp47:collagen) at OD600 values (*n* = 3 data point representing mean value of technical triplicates of each experiment with error bars representing standard deviation).

Hsp47 has been shown to prevent collagen fibrillogenesis in vitro. Previous reports have demonstrated that addition of Hsp47 in twofold molar excess to a 0.6 × 10^−6^ m collagen solution in PBS delays collagen fibrillation at 34 °C.[[qv: 13b,26]] Similar fibrillation assays performed with H_47N_ solutions using turbidity measurements reproduced these results (see Figure S3 in the Supporting Information). When using minimum essential medium (MEM) for the experiments, improved gelation was observed, and confirmed by rheology measurements (see Figure S4 in the Supporting Information). MEM is considered more representative of physiological conditions for collagen association^27^ and was used for further fibrillation assays with Hsp47 variants at concentrations between 0.1 × 10^−6^ and 1.2 × 10^−6^ m. H_47Y<ONBY_, H_47Y<R_ and EGFP did not show any effect on fibrillation kinetics of collagen solutions at any tested concentration (Figure 2c). Light‐activated H_47Y<ONBY_ *_hv_* reduced the rate of collagen fibrillation to a similar extent to H_47N_ at comparable concentrations. These results indicate that H_47Y<ONBY_ *_hv_* enables light‐triggered interference with lateral association of collagen triple helices and delay of fibril formation.

### 2.3 Hsp47 Variants Can Be Delivered into ER via KDEL Receptor‐Mediated Endocytosis

Hsp47 is an ER resident protein with a C‐terminal KDEL retention motif. This motif is recognized by KDEL receptor after Hsp47 release in the Golgi and is responsible for its retention in the ER.^28^ In fact, deletion of KDEL sequence has been shown to block the retention of Hsp47 into the ER.^29^ The KDEL receptor is also present in the plasma membrane of cells, and has been shown to assist internalization of KDEL containing molecules from the extracellular space.^30^ We tested if our Hsp47 variants could be delivered to ER using KDEL receptor‐mediated endocytosis (**Figure** **3**). For this purpose, L929 and MEFs fibroblasts were incubated with Hsp47 variants for 3 h and imaged. Interestingly, cells incubated with H_47N,_ H_47Y<R_, and H_47Y<ONBY_ *_hv_* showed colocalization of the EGFP signal (green in Figure 3) with the ER tracker dye (red), indicating successful uptake of the Hsp47 variant (see 10×‐magnified images in Figure S7 in the Supporting Information). Neither uptake of the H_47KDEL_ variant with deleted KDEL, nor uptake of EGFP was observed after 3 h incubation. In order to optimize the Hsp47 concentration for efficient delivery to fibroblast cells, experiments with concentrations of H_47N_ in the incubation medium between 0.01 × 10^−6^ and 1 × 10^−6^ m were performed. 0.2 × 10^−6^–0.3 × 10^−6^ m concentration proved to be the best condition for the delivery of the recombinant constructs (see Figure S6 in the Supporting Information). Protein concentrations above 0.3 × 10^−6^ m resulted in the formation of protein aggregates on the cell culture substrate. These results demonstrate that the photoactivatable H_47Y<ONBY_ *_hv_* can be simply introduced into the ER of cells by short incubation, allowing easy experimental implementation of this tool for the study of Hsp47‐specific roles in cellular pathways and collagen assembly.

**Figure 3:** Photoactivatable Hsp47 delivery to ER via KDEL receptor‐mediated endocytosis. Confocal Z stack images of L929 cells after incubation with Hsp47 variants showing colocalization of H_47N_ or H_47Y<ONBY_ signal and ER staining. No fluorescence was observed after incubation with EGFP or H_47KDEL_ constructs (blue: DAPI (Nucleus), Green: EGFP (Hsp47 variants), and Red: ER tracker dye); scale bar: 10 µm.

### 2.4 Increase in Collagen Production in Hsp47 −/− Cell Cultures in Response to Photoactivation of H_47Y<ONBY_

Collagen biosynthesis is dependent on the expression level of functional Hsp47. To determine the bioactivity of up taken Hsp47 variants, we investigated collagen biosynthesis of Hsp47 −/− cells after incubation with the recombinant proteins. The deposited collagen was quantified using the Sirus Red assay, whose dye binds specifically to the [Gly‐*X*‐*Y*] *n* helical structure on fibrillar collagen types I to V.[[qv: 17a]] Hsp47 −/− cells incubated with H_47N_ showed a significant increase in collagen production (≈15–20%). Hsp47 −/− cells incubated with H_47Y<ONBY_ did not show increase in collagen production, in agreement with the lack of biofunctionality of H_47Y<ONBY_ observed in previous experiments. Exposure of H_47Y<ONBY_ treated cells with 405 nm light in situ lead to an increase in collagen production. Within the concentration range used (estimated as H_47Y<ONBY_ 0.012 × 10^−9^ m per cell) no cytotoxicity effect was observed (Figure S11, Supporting Information). Note that the ONB photoremovable group has been used in in vitro and in vivo^24^, ^31^ applications and no significant cytotoxicity associated with the released photoproduct could be detected. These results demonstrate biofunctionality of H_47Y<ONBY_ intracellularly in response to light activation (**Figure** **4**b). Ascorbate (vitamin C) is a widely used chemical inducer for collagen production at translational level by triple helix stabilization.^32^ We compared collagen deposition in Hsp47 −/− cells treated with H_47N_, with light exposed H_47Y<ONBY_ and with ascorbate. Interestingly, we found higher levels of collagen production in H_47N_ and light exposed H_47Y<ONBY_ incubated cells compared to ascorbate treated cells (Figure 4b). Addition of ascorbate to cells containing H_47N_ or light exposed H_47Y<ONBY_ *_hv_* had a synergistic effect for collagen production (see Figure 4c). When Hsp47 +/+ cells were treated with H_47N_ or with in situ activated H_47Y<ONBY_ *_hv_* only a slight increase in collagen production was observed (see Figure 4c). However, H_47N_ caused a change in cell morphology: enhanced spreading was observed (Figure S9, Supporting Information). Interestingly, proliferation levels in Hsp47 −/− cultures treated with H_47N_ or in situ activated H_47Y<ONBY_ were higher than in nontreated cultures (see Figure S5 in the Supporting Information). Together, these results demonstrate the efficiency of exogenous H_47<ONBY_ to upregulate collagen biosynthesis upon light exposure in Hsp47 −/− cells, and to enhance cell spreading in Hsp47 +/+ cells (Figure 4).

**Figure 4:** Stimulated collagen deposition using photoactivatable Hsp47. a) Scheme showing photoactivation of H_47Y<ONBY_ and stimulated collagen deposition in Hsp47 deficient cells. b) Relative collagen deposition in Hsp47 +/+ and Hsp47 −/− cultures treated with Hsp47 variants and ascorbate. c) Relative collagen deposition in Hsp47 +/+ and Hsp47 −/− cultures treated with Hsp47 variants with or without ascorbate. Collagen deposition was calculated using quantified data of Sirus Red Assay at 570 nm (*n* = 3 data point representing mean value of technical triplicates of each experiment with whisker plots representing standard deviation). Statistical significance was analyzed by Tukey test, which shows significant differences between conditions. Significance was calculated by comparing Hsp47 +/+ to Hsp47 −/− and on photoactivation of H_47Y<ONBY_ delivered in Hsp47 −/− (mean ± SD, ANOVA, *** *p* < 0.001).

### 2.5 Controlled Light Exposure Allows Spatial Regulation of Collagen Production

Finally, we investigated the potential of H_47Y<ONBY_ for spatiotemporal control of collagen production after in situ photoactivation of cell cultures. For this purpose, an assay for imaging collagen deposition on the culture substrate was established. Hsp47 −/− cells were incubated with the different Hsp47 variants for 3 h. Then the medium was exchanged and cells were cultured for further 24 h, fixed, and stained with Col1 Antibody for imaging deposited collagen type I on the culture substrates. Hsp47 −/− cells incubated with H_47Y<R_, H_47KDEL_ or EGFP did not show any fluorescence signal, whereas cells incubated with H_47N_ showed a clear fluorescence corresponding to collagen production (**Figure** **5**b). H_47N_ and light exposed H_47Y<ONBY_ showed EGFP fluorescence located at the ER, indicating that the recombinant protein delivered was still present intracellularly after 24 h (Figure 5). This is in agreement with the reported >24 h half‐life of Hsp47.^33^ H_47Y<R_ did not show EGFP fluorescence after 24 h, which may be due to degradation because of lack of functional activity over time (Figure 5b). Altogether these results demonstrate that H_47Y<ONBY_ can be used in cell cultures to increase collagen production at a selected time point. In order to test the spatial resolution of the light‐induced collagen deposition,1.8 × 1.2 mm^2^ areas of the Hsp47 −/− cell culture previously incubated with H_47Y<ONBY_ were irradiated for 30 sec at 405 nm an hour after medium exchange. Higher dose results in cell damage.^33^ Cells at the exposed areas showed significant higher collagen deposition (Figure 5a). Hsp47 −/− and Hsp47 +/+ cells lacking exogenous H_47Y<ONBY_ did not show any increase in collagen staining upon exposure, indicating that UV irradiation by itself had no effect on collagen production (Figure 5).

**Figure 5:** Localized induction of collagen deposition by photoactivation of photoactivatable Hsp47. Immunostaining of MEF Hsp47 +/+ and −/− cultures 24 h after treatment with different Hsp47 variants and controls Col1 antibody staining in red, Hsp47 variants in green (EGFP), and nuclei in blue (DAPI). a) Hsp47 +/+ and −/− having no protein delivery were used as controls. The light exposed areas (1.8 × 1.2 mm^2^) are highlighted with dotted square. Irradiation wavelength was 405 nm. b) Hsp47 +/+ cells incubated with other inactive mutants did not show enhanced collagen production, whereas cells incubated with H_47N_ showed higher collagen levels. Scale bar: 250 µm.

In order to evaluate the spatial accuracy of the photoinduced collagen deposition in Hsp47 −/− cells treated with H_47Y<ONBY_, independent 1.13 mm^2^ areas of the culture were scanned at 405 nm. We observed increased collagen deposition within the exposed areas after staining with collagen I antibody (Figure S13, Supporting Information). In addition, cells within the scanned area showed a different morphology (Video 1, Supporting Information). These results demonstrate the possibility to use H_47Y<ONBY_ to photoregulate collagen biosynthesis in cell cultures and build spatially defined collagen networks.

## 3 Conclusion

A photoactivatable variant of the collagen‐specific protein Hsp47 has been developed by incorporating a photoactivatable Tyr rest at the 383rd amino acid of Hsp47, which is relevant for collagen binding. This recombinant protein could be effectively delivered to the ER of fibroblasts via KDEL receptor‐mediated endocytosis. In situ light exposure allowed light‐mediated increase of functional Hsp47 concentration inside the cells, and consequently localized upregulation of collagen production and deposition in cellular cultures. Therefore, we speculate this tool would also be useful in studies or applications in those cells which normal levels of Hsp47. We envision that this tool will allow unprecedented studies of collagen synthesis and early assembly. Photoactivation at submicron level will allow precise control and simultaneous monitoring of collagen‐related intracellular events. Moreover, photoactivatable Hsp47 might inspire new therapeutic concepts for treating collagen‐related defects like osteogenesis imperfecta, Ehlers–Danlos syndrome, and epidermolysis bullosa by promoting correct folding of collagen. Finally, the possibility of external upregulation of collagen synthesis and deposition might be advantageous for tissue regeneration and rebuilding of the extracellular scaffold.

## Conflict of Interest

The authors declare no conflict of interest.

## Supporting information

Supplementary
